# Multiple Performance Evaluation of Bionic Thin-Walled Structures with Different Cross Sections considering Complex Conditions

**DOI:** 10.1155/2022/2220633

**Published:** 2022-09-29

**Authors:** Honghao Zhang, Zhongwei Huang, Tao Li, Chonghua Bao, Liang Zhang

**Affiliations:** ^1^Key Laboratory of High Efficiency and Clean Mechanical Manufacture (Ministry of Education), School of Mechanical Engineering, Shandong University, Jinan 250061, China; ^2^Key Laboratory of Traffic Safety on Track of Ministry of Education, School of Traffic and Transportation Engineering, Central South University, Changsha 410000, China; ^3^Joint International Research Laboratory of Key Technology for Rail Traffic Safety, Central South University, Changsha 410000, China; ^4^Chongqing Key Laboratory of Vehicle Crash/Bio-Impact and Traffic Safety, Institute for Traffic Medicine, Daping Hospital, Army Medical University, Chongqing 400000, China

## Abstract

Bionic thin-walled structures, due to their excellent energy absorbing capacity, low manufacturing cost, and remarkable level of lightweight, have been widely applied in the field of traffic safety protection. Combinatorial structures that incorporate the prototypical characteristics of multiple organisms also turn into the hotspot of the research on safety protection structure, which can achieve more excellent overall performance. However, how to select the optimal alternative considering the performance of different attributes and different accident conditions has become an urgent problem to be solved. This paper proposes 12 kinds of bionic thin-walled energy absorption structures with different cross sections and bamboo of tubes, which is inspired by the structural characteristics of bamboo. A comprehensive performance analysis, including specific energy absorption, peak crushing force, and undulation of the load-carrying capacity under quasi-static and dynamic conditions, is carried out based on the finite element simulation. The gray relational analysis method is applied to select the optimal structure. In addition, sensitivity analysis of each structural variable is conducted. The result shows that the “+-3” bionic thin-walled structure has the best comprehensive performance, and the structural variable has great impact on the *PCF*. This study provides an effective decision-making support tool for performance evaluation of bionic thin-walled structures.

## 1. Introduction

In passive safety design of automobile, thin-walled structure has been widely used as energy absorption device due to their excellent energy absorbing capacity, low manufacturing cost, and remarkable level of lightweight [1–3]. Single-walled structures and multicell structures have been extensively in recent years by theoretical derivation, experimental testing, numerical simulation, and multidisciplinary optimization [4–7].

Bionic thin-walled structures [8, 9], which are inspired by the design principles of natural structures, have recently attracted wide attention to achieve better crashworthiness and lightweight level, e.g., beetle-inspired structures [10, 11], woodpecker-inspired structures [12, 13], mantis shrimp-inspired structures [14, 15], and shrimp chela structures [16]. For example, Du et al. proposed a novel thin-walled energy absorption structure with hollow columns by studying the beetle elytra [17]. Zhang et al. conducted a systematic review on various biological systems with sophisticated architectures perfectly for impact resistance and energy absorption and conduct dynamic behaviors analysis of each structure from the perspective of design, mechanisms, and models [18]. Wu et al. proposed a novel bionic tree-like fractal structure, which is applied as energy absorber under axial loading, and analyze the ability of energy absorption under quasi-static and dynamic conditions [19]. Ha et al. proposed a novel bio-inspired fractal multicell circular tubes for energy absorption and conducted crashworthiness analysis of multicell circular tubes under axial crushing [20]. In addition, the geometric fractal and hierarchical structural designs have also been incorporated into the design of energy-absorbing structures to achieve higher mechanical properties. However, how to select the optimal alternative considering the performance of different attributes and different accident conditions has become an urgent problem to be solved. Many scholars introduce the multiple attribute decision-making (MADM) method into optimization of energy absorption structure. However, compared with other MADM methods, the gray relationship analysis (GRA) method can consider the shape similarity of every alternative to make the overcome more reliable. Vinayagar et al. used the Taguchi method and combines the gray relationship analysis to analyze the parameters affecting the crash resistance characteristics of the double-tube structure and determine the optimal crash tolerance parameters [21]. Yu analyzed the performance structure satisfying the functional classification of the Pareto front solutions [22]. Zhang proposed a hybrid optimization method based on best worst method (BW) and GRA to solve the train energy absorption structure optimization and then to find the optimal energy absorption parameters [23]. Wang introduces a multicriterion decision approach combining integrated entropy and GRA method to find an ideal balance between the energy absorption (EA) and the initial peak breaking force (IPCF) [24].

Based on the correlation analysis as described above, this paper proposes a hybrid decision-making method of multiple performance evaluation of bionic thin-walled structures. The main highlights of the research are summarized as follow: (1) 12 kinds of bionic thin-walled energy absorption structures with different cross sections and hierarchies of tubes are simulated and analyzed, which is inspired by the structural characteristics of bamboo and horsetail; (2) a comprehensive performance analysis, including specific energy absorption (*SEA*), peak crushing force (*PCF*), and undulation of the load-carrying capacity (*ULC*), is carried out under quasi-static and dynamic conditions; and (3) the GRA method is applied to select the optimal structure and sensitivity analysis of each structural variable is conducted.

The rest of this paper is organized as follows. In Section 2, structural description of 12 kinds of bionic thin-walled energy absorption structures with different cross sections and hierarchies of tubes is conducted.  Section 3 carries out the performance analysis and evaluation of bionic thin-walled structures. Sensitivity analysis of structural parameters is conducted in Section 4. The last section concludes this work.

## 2. Structural Description

### 2.1. Geometrical Design

Since ancient times, China has praised for the tenacity of bamboo, which is closely related to its own excellent structural characteristics. In nature, after continuous evolution and deduction, the structural changes of living organisms tend to resist the harsh living environment, which show good mechanical characteristics. Zou et al. [25] found that moso bamboo growing for one year is 1.85 times stronger than that of 2A12 aluminum alloy because of its special lightweight characteristic. Its complex hollow cylindrical structure showing good mechanical properties has attracted the attention of many researchers [26]. The structure, load, and function of bamboo are very similar to those of thin-walled tubes, so the bionic thin-walled tubes of bamboo are increasingly studied.

Bamboo is a plant with a hollow structure separated by a solid transverse diaphragm along the length direction of the pole [27]. The bamboo cross section is irregular round, and the stem wall surrounded by the inner layer and the outer epidermis presents a double ring structure, such a structure is conducive to protect the tissue. This special tubular structure can withstand all kinds of shocks and damage from bad weather. A series of thin-walled cells composed of different shaped ribs can have important effects on the axial mechanical properties of bamboo stems. Liu et al. [28] found that the interaction between rib and tube has a significant effect on its collision tolerance. Therefore, many researchers draw on the bamboo structure and propose some different new cylindrical bionic structures of the rib plate. Although many researchers have designed the cross section of the imitation bamboo structure, the performance comparison and its structure optimization are lacking.

In this study, 12 structures with four types of cross sections and three types of hierarchies of tubes are designed, as shown in Figure 1. Bionic tube parameters are set as follows: test height (*h*) =160 mm, outer circle diameter (*D*) =90 mm, inner circle diameter (*d*) =60 mm, outer circle thickness (*t*_1_) = 1 mm, inner circle thickness (*t*_2_) = 1 mm, small circle thickness (*t*_3_) = 1 mm, and rib shape thickness (*t*_4_) = 1 mm [19, 29].

### 2.2. Finite Element Model of Bionic Thin-Walled Structures

The finite element model of bionic thin-walled structures is constructed by LS-DYNA software, which is shown in Figure 2. In this model, the center diameter of the rib plate is set to 50 mm, the angle of the rib plate is set to 45°, and the thickness of the rib plate is set to 1 mm. In addition, the bionic circular tube diameter, thickness, and length are set to 62 mm, 1 mm, and 100 mm, respectively. The bottom end of the bionic tube is fixed to the ground, and the rigid wall compresses the bionic circular tube at a constant speed of 10 m/s to 75% of the initial length. The bionic circular tube adopts thin shell unit and grid size is 1 mm × 1 mm. The compression deformation scheme is shown in Figure 3.

Numerical simulation adopts two types of contact methods. The contact surface of the bionic circular tube and the rigid wall is modeled using the “automatic face-to-face” contact algorithm. Considering the contact of the bionic circular tube wall during folding, an “automatic monolithic” contact algorithm is established. The static and dynamic friction coefficient in the defined contact is 0.2 [30].

The Mat 123 material model in LS-DYNA is applied to define the aluminum alloy (6063T5), and the mechanical properties of the material are tested [29]. The parameters of 6063T5 material are shown in Table 1. Because aluminum alloy is not sensitive to strain rate, the strain rate effect is not considered [31]. The comparison and verification results of finite element simulation are shown in Figure 4. The error is less than 4%, which proves the validity of finite element simulation.

## 3. Performance Analysis and Evaluation of Bionic Thin-Walled Structures

### 3.1. Performance Metrics

To evaluate the performance of bionic circular tubes, the following indicators of crashworthiness are introduced [32–34].

The EA represents the total energy absorbed within the effective impact distance.

(1) $$\begin{array}{c} \text{EA}=\int_{0}^{d}F\left(x\right)\text{dx }, \end{array}$$

where *d* indicates the compression displacement and *F*(*x*) indicates the crush force value during the deformation.The *SEA* represents the energy dissipation per unit mass, which is an important index to evaluate the collision resistance of energy absorption structure.

(2) $$\begin{array}{c} \text{SEA}=\frac{\text{EA}}{m}, \end{array}$$

where *m* represents the mass of the bionic circular tube.

The *PCF* represents the maximum force received during the impact, which can usually represent the survival rate of the passengers in the train. The *PCF* represents the peak force in the load-displacement curve of an energy absorber, often corresponding to the formation of the first fold. This value should be within a tolerance limit to crushing. The mean crushing force (*MCF*) is defined as total energy absorption divided the corresponding displacement, as shown in

(3) $$\begin{array}{c} \text{MCF}=\frac{\text{EA}\left(d\right)}{d}. \end{array}$$

Collision force efficiency (*CFE*) indicates the load stability of the energy absorption structure. The larger the value indicates the greater the stability during the collision process.

(4) $$\begin{array}{c} \text{CFE}=\frac{\text{MCF}}{\text{PCF}}. \end{array}$$

The *ULC* is calculated as

(5) $$\begin{array}{c} \text{ULC}=\frac{\int_{0}^{d}\left|F\left(x\right)-\text{MCF}\right|}{\text{EA}}. \end{array}$$

### 3.2. Performance Analysis under Quasi-Static and Dynamic Conditions

The bionic thin-walled energy-absorbing structures is applied to the train collision working condition, and *EA*, *PCF*, and *ULC* of different rib structures are compared in the same working condition. The axial shock scheme of the bionic circular tube as shown in Figure 5 and the LS-DYNA are applied to simulate the collisions of the energy-absorbing structure. Bionic circular tubes are constrained by six degrees of freedom at the bottom to prevent any translational or rotational motion. The specified uniform working condition is that the top of the bionic circular tube is impacted by a rigid wall with a mass of 500 kg at an initial speed of 10 m/s. The quasi-static condition is 6.66 mm/min. The bionic circular tube adopts the thin shell unit, the grid size is 2 mm × 2 mm, and the material of rigid wall uses the rigid material Mat 20 in LS-DYNA.

Numerical simulation adopts two types of contact methods. The contact surface of the bionic circular tube and the rigid wall is modeled using the “automatic face-to-face” contact algorithm. Considering the contact of the bionic circular tube wall during folding, an “automatic single side” contact algorithm is established. The static friction coefficient in the defined contact is 0.3, and the dynamic friction coefficient is 0.2. Bionic circular pipe material is made of aluminum alloy (AA6061-O) and defined by the Mat 24 material model in LS-DYNA. The material mechanical properties of aluminum alloy AA6061-O are shown in Table 2 [35]. Because aluminum alloy is not sensitive to strain rate, the strain rate effect is not considered [35].

When the collision process is simulated under the same operating conditions, *EA*, *PCF*, and *ULC* of the 12 models at the compression time of from 75% to 120 mm are output, as shown in Table 3 and Figure 6.

According to the data analysis in Tables 2–4, the following conclusions can be obtained: (1) the influence of the cross-section shape on *SEA*, *PCF*, and *CFE* is obviously different, and (2) the *SEA* and *PCF* of the model are contradictory. When the *SEA* is the best, the performance of *PCF* is not good. The larger the structural order, the larger *SEA*, the greater *PCF*, and the smaller the *ULC*. (3) The level 3 structures *ULC* and *SEA* have a large advantage, and *PCF* is slightly not superior.

### 3.3. Multiple Performance Evaluation

In this subsection, the GRA method is applied to select the optimal structure [36]. Note that the value of the gray relational closeness indicator, i.e., *R*, is expected to be as large as possible to get closer to the best performance. The results of multiple performance evaluation can be calculated by GRA method, as shown in Figure 7.

According to the results of Figure 7, the final rank of 12 kinds of bionic thin-walled energy absorption structures can be obtained, i.e., +-3> + -2> + -1>H-2>T-3>O-2>O-3>T-2>T-1>H-3>O-1>H-1. Thus, the “+-3” structure has the best comprehensive performance.

## 4. Analysis

The crashworthiness response is closely related to the geometry and material distribution of thin-walled structures. In this section, the “+ -3” structure is selected as the research object, which has better collision resistance properties, to get a comprehensive understanding of the effects of different parameters on crashworthiness.

### 4.1. Effect of the Inner Circle Radius to the Crashworthiness

The size of the inner circle radius determines the geometric properties of the structure. Therefore, this section explores the effect of the *r* on the crashworthiness of the “+-3” structure. Due to geometric limitations, the range of *r* is set to 50 mm to 70 mm. Wall thickness and fragmentation displacement are 1 mm and 120 mm, respectively.

The results of *SEA*, *PCF*, and *ULC* with different *r* are shown in Table 4 and Figure 8. With increasing *r*, both *SEA* and *PCF* decreased, and *PCF* decreased significantly, and the *ULC* is distinguished less between 50 mm and 66 mm, but the *ULC* shows an upward trend after *r* > 66 mm. The results show that the *PCF* is most affected by the size of the inner circle radius, and the *PCF* decreased with increasing *r*. Since the *SEA* and *ULC* changes are not obvious, increasing the radius of the inner circle is beneficial to improve the crashworthiness of the “+-3” structure.

### 4.2. Effect of the Outer Circle Thickness to the Crashworthiness

The change of the outer circle thickness determines the geometric properties of the structure. Therefore, this section explores the effect of the *t*_1_ on the crashworthiness. Due to geometric limitations, the range of *r* is set to 0.5 mm to 1.5 mm. Wall thickness and fragmentation displacement are set to 1 mm and 120 mm, respectively.

The results of *SEA*, *PCF*, and *ULC* with different *t*_1_ are shown in Table 5 and Figure 9. With the increase of *t*_1_, little obvious trends in *SEA* and *ULC*, the *PCF* increased linearly with increasing *t*_1_. The analysis shows that the *t*_1_ change has no effect on the improvement of *SEA* and *ULC* but has a greater effect on *PCF*. Thus, as the thickness of the outer circle increases, the crashworthiness of the “+-3” structure is reduced.

### 4.3. Effect of the Inner Circle Thickness to the Crashworthiness

The change of the inner circle thickness determines the geometric properties of the structure. Thus, this section explores the effect of the *t*_2_ on the crashworthiness of the “+-3” structure. Due to geometric limitations, the range of *t*_2_ is set to 0.5 mm to 1.5 mm. Wall thickness and fragmentation displacement are 1 mm and 120 mm, respectively.

The results of *SEA*, *PCF*, and *ULC* with different *t*_2_ are shown in Table 6 and Figure 10. With the increase of *t*_2_, little obvious trends in *SEA* and *ULC*, the *PCF* increased linearly with increasing *t*_2_. The analysis shows that the *t*_2_ change has no effect on the improvement of *SEA* and *ULC* but has a greater effect on *PCF*. Thus, as the thickness of the inner circle increases, the crashworthiness of the “+-3” structure is reduced.

### 4.4. Effect of the Small Circle Thickness to the Crashworthiness

The change of the small circle thickness determines the geometric properties of the structure. Therefore, this section explores the effect of the *t*_3_ on the “+-3” structure crashworthiness. Due to geometric limitations, the range of *t*_3_ is set to 0.5 mm to 1.5 mm. Wall thickness and fragmentation displacement are 1 mm and 120 mm, respectively.

The results of *SEA*, *PCF*, and *ULC* with different *t*_3_ are shown in Table 7 and Figure 11. With the increase of *t*_3_, the *SEA* and *PCF* show a gradually rising trend, and the *ULC* shows a downward trend. The analysis of the results shows that more *t*_3_ affects *PCF* than *SEA* and *ULC*, and the increase of the small circle thickness is beneficial to improve the crashworthiness of the “+-3” structure.

### 4.5. Effect of the Cross Thickness to the Crashworthiness

The change of the cross thickness determines the geometric properties of the structure. Therefore, this section explores the effect of the *t*_4_ on the crashworthiness of the “+-3” structure. Due to geometric limitations, the range of *t*_4_ is set to 0.5 mm to 1.5 mm. Wall thickness and fragmentation displacement are 1 mm and 120 mm, respectively.

The results of *SEA*, *PCF*, and *ULC* with different *t*_4_ are shown in Table 8 and Figure 12. With the increase of *t*_4_, the *SEA* and *PCF* show a gradually rising trend, and the *ULC* shows a downward trend. The analysis of the results shows that more *t*_4_ affects *PCF* than *SEA* and *ULC*, and the increase of the cross thickness is beneficial to improve the crashworthiness of the “+-3” structure.

## 5. Conclusion

The demand for lightweight structures with high-energy absorption capacity is increasing in aerospace, transport, and train transport. In this study, we constructed the wall structure of horsetail and bamboo and performed finite element simulation under quasi-static and dynamic conditions. The study designs 12 train energy absorption structures and uses the GRA decision method to select the optimal energy absorption structure that is “+-3”. And the collision resistance of “+ -3” with different structure parameters, such as *SEA*, *PCF*, and *ULC*, is also analyzed to obtain the train energy absorption structure with the best collision performance. The result shows that the structural parameters, including inner circle radius, outer circle thickness, inner circle thickness, small circle thickness, and cross thickness, have great impact on the performance of *PCF*, and have little effect on other performances. This study provides an effective decision-making support tool for performance evaluation of bionic thin-walled structures.

In future research, our works will focus on (1) proposing more advanced decision-making methods to select optimal alternative [37, 38] and (2) by noting that the raw data have the features of indirectness, indefiniteness, and fuzziness, integrating cloud model theory or fuzzy theory into the MADM method for further development [39].

## Figures and Tables

**Figure 1:** 12 structures of bionic tube cross section.

**Figure 2:** Finite element model of thin-walled structure.

**Figure 3:** Compression scheme.

**Figure 4:** Force-displacement curve comparison diagram.

**Figure 5:** Axial impact scheme.

**Figure 6:** Performances of the different energy-absorbing structures.

**Figure 7:** The results of multiple performance evaluation.

**Figure 8:** *SEA*, *PCF*, and *ULC* with different *r*.

**Figure 9:** *SEA*, *PCF*, and *ULC* with different *t*_1_.

**Figure 10:** *SEA*, *PCF*, and *ULC* with different *t*_2_.

**Figure 11:** *SEA*, *PCF*, and *ULC* with different *t*_3_.

**Figure 12:** *SEA*, *PCF*, and *ULC* with different *t*_4_.

**Table 1:** The characteristics parameters of 6063T5 material.

Aluminum alloy attribute	Symbol	6063T5 [5]
		Mat 123
Yield stress (MPa)	*σ*_*Y*_	179.67
Ultimate strength (MPa)	*σ*_*μ*_	241.83
Elongation (%)	*e*_*b*_	9.98
Elasticity modulus (GPa)	*E*	68.50
Density (g/cm^3^)	*ρ*	2.70
Poisson ratio	*μ*	0.33

**Table 2:** The characteristics parameters of AA6061-O material.

Aluminum alloy attribute	Symbol	Value
Density	*ρ*	2.7 × 10^3^ kg/m^3^
Young modulus	*E*	68.2 Gpa
Poisson ratio	*ν*	0.3
Initial yield stress	*σ*_*y*_	96.6 Mpa
Ultimate strength	*σ*_*u*_	194.3 Mpa

**Table 3:** Performances of 12 models under quasi-static and dynamic conditions.

Quasi-static	*SEA*/(J/kg)	*PCF*/kN	*ULC*	Dynamic	*SEA*/(J/kg)	*PCF*/kN	*ULC*
O-1	11970.60235	48.26073074	0.129895495	O-1	15297.53364	73.02017975	0.281920234
O-2	19798.69752	73.36416626	0.078820047	O-2	23067.38316	97.48590088	0.136284609
O-3	23035.2155	88.81903076	0.067117202	O-3	26022.71119	116.0002289	0.09034401
+-1	13216.34816	44.27799988	0.095279724	+-1	16926.01061	71.81346893	0.173698935
+-2	16997.07670	58.50913239	0.074431542	+-2	20185.7341	81.74725342	0.142577882
+-3	26024.56077	94.06425476	0.042442561	+-3	27818.25861	116.0982819	0.073220433
T-1	11967.14202	44.09593582	0.079961108	T-1	15764.99293	79.57016754	0.21101312
T-2	18177.65906	72.82758331	0.082018615	T-2	21643.22482	95.43017578	0.156808657
T-3	25097.9928	98.97866821	0.049341720	T-3	27308.82226	121.3243027	0.077072887
H-1	14582.77206	50.90706253	0.154837602	H-1	17582.58251	85.42107391	0.258364411
H-2	21740.24771	71.87575531	0.079805126	H-2	23650.37544	93.50915527	0.144775426
H-3	25130.57754	105.0628662	0.085302177	H-3	27865.90662	127.355896	0.080808509

**Table 4:** *SEA*, *PCF*, and *ULC* with different *r*.

*r* (mm)	*SEA*	*PCF*	*ULC*
50	27753.47397	123.5179749	0.067473139
54	27908.04172	121.4720688	0.070847867
58	27847.74066	118.0526733	0.064985456
62	27847.06597	114.9915924	0.066431703
66	27735.90969	110.8166733	0.066782156
70	26209.21827	109.7163925	0.104511352

**Table 5:** *SEA*, *PCF*, and *ULC* with different *t*_1_.

*t*_1_ (mm)	*SEA*	*PCF*	*ULC*
0.5	28110.81729	94.90704346	0.080366043
0.7	28374.95199	103.7966690	0.063082608
0.9	27990.96810	112.0767822	0.078752285
1.1	27925.79211	120.847023	0.066761015
1.3	28252.12913	129.6835327	0.065778083
1.5	28206.08269	138.2976379	0.077431486

**Table 6:** *SEA*, *PCF*, and *ULC* with different *t*_2_.

*t*_2_ (mm)	*SEA*	*PCF*	*ULC*
0.5	27462.99004	102.3353119	0.079881044
0.7	27393.21828	108.0727158	0.069060377
0.9	27450.81637	113.4499359	0.072175099
1.1	28537.44656	118.6362915	0.068084331
1.3	28095.03258	124.4785919	0.076911615
1.5	29293.74905	130.1577759	0.074497454

**Table 7:** *SEA*, *PCF*, and *ULC* with different *t*_3_.

*t*_3_ (mm)	*SEA*	*PCF*	*ULC*
0.5	25272.0107	103.4063721	0.090000038
0.7	26735.35855	108.2516480	0.082480691
0.9	27398.05367	113.3823547	0.079303618
1.1	28603.43736	118.8743744	0.065200003
1.3	29693.61150	124.1996613	0.062803206
1.5	30479.45914	128.7521973	0.069161248

**Table 8:** *SEA*, *PCF*, and *ULC* with different *t*_4_.

*t*_4_ (mm)	*SEA*	*PCF*	*ULC*
0.5	26132.48097	107.3699265	0.087749405
0.7	26790.31066	110.7307739	0.079431924
0.9	27520.00703	114.3213196	0.062160811
1.1	28262.00177	117.868782	0.069857864
1.3	29283.03848	121.7102356	0.074257387
1.5	30177.41526	125.7415619	0.056119828

## Data Availability

The study did not report any data.
